The article "Analysis of the Effect of Laparoscopic Cholecystectomy for Acute Cholecystitis after Percutaneous Transhepatic Gallbladder Puncture and Drainage" was retracted in 2023. Reasons: signs of a paper mill; compromised peer review; unreliable results or conclusions.

# Analysis of the Effect of Laparoscopic Cholecystectomy for Acute Cholecystitis after Percutaneous Transhepatic Gallbladder Puncture and Drainage

**DOI:** 10.1155/2022/2071326

**Published:** 2022-07-20

**Authors:** Jia-Peng Yang, Zhong Tian

**Affiliations:** Department of General Surgery, Shengjing Hospital of China Medical University, Shenyang 110004, Liaoning Province, China

## Abstract

**Objective:**

To assess the effect of laparoscopic cholecystectomy for acute cholecystitis after percutaneous transhepatic gallbladder drainage (PTGBD).

**Methods:**

A total of 70 patients with acute cholecystitis diagnosed and treated in our hospital between April 2020 and November 2021 were recruited and assigned to receive either conventional treatment (conventional group) or PTGBD plus laparoscopic cholecystectomy (experimental group) according to the order of admission (with January 2021 as the cut-off time point), with 35 cases in each group. Outcome measures included treatment outcomes, surgical indices, and postoperative recovery.

**Results:**

Patients in the experimental group showed significantly less intraoperative hemorrhage volume and shorter operative time, time-lapse before passing gas, and hospital stay (83.15 ± 31.17, 32.54 ± 12.61, 23.02 ± 4.61, 7.98 ± 3.24) versus those in the conventional group (120.56 ± 30.55, 61.01 ± 15.54, 28.15 ± 5.91, 11.95 ± 4.15) (*P* < 0.05). The incidence of conversion to open surgery and postoperative drainage in the experimental group was significantly lower (2.86%, 5.71%) than that of the conventional group (25.71%, 45.71%) (*P* < 0.05). The differences in the postoperative body temperature of the two groups did not come up to statistical standard (*P* > 0.05). The experimental group had faster body temperature recovery and leukocyte recovery and better leukocyte levels (1.25 ± 0.56, 2.36 ± 0.48, 7.92 ± 1.36) than the conventional group (3.11 ± 1.05, 5.41 ± 0.63, 10.52 ± 2.78) (*P* < 0.05). There was 1 (2.86%) case of pneumothorax and 1 (2.86%) case of intestinal bleeding in the experimental group, and there were 2 (5.71%) cases of biliary leakage, 3 (8.57%) cases of pneumothorax, 4 (11.43%) cases of intestinal bleeding, 5.71% cases of incisional infection, 1 (2.86%) case of respiratory failure, and 1 (2.86%) case of liver damage in the conventional group. The experimental group showed a significantly lower incidence of complications (5.71%) versus the conventional group (37.14%) (*P* < 0.05).

**Conclusion:**

PTGBD plus laparoscopic cholecystectomy for acute cholecystitis effectively improves surgical safety, promotes patients' postoperative recovery, and reduces the incidence of conversion to open surgery and postoperative complications with a high safety profile. Further trials are, however, required prior to clinical promotion.

The article "Analysis of the Effect of Laparoscopic Cholecystectomy for Acute Cholecystitis after Percutaneous Transhepatic Gallbladder Puncture and Drainage" was retracted in 2023. Reasons: signs of a paper mill; compromised peer review; unreliable results or conclusions.

## 1. Introduction

Acute cholecystitis is a common acute gastrointestinal disorder caused by obstruction of the bile cyst duct and bacterial invasion. Clinical data show that its incidence is only second to acute appendicitis [1, 2]. Its main clinical manifestation is paroxysmal colic in the right upper abdomen with significant tenderness and abdominal stiffness, and the pain may extend to the right shoulder and back. Acute cholecystitis is an acute inflammatory disease with typical inflammatory manifestations of redness, swelling, pain, and dysfunction. Because the gallbladder is deep in the abdomen, local signs and symptoms, such as fever (mild to moderate) and rapid heartbeat, occur when gallbladder inflammation spreads to the peritoneum. However, the presence of chills or high fever is indicative of a serious condition [3, 4]. Relevant epidemiological statistics show that acute cholecystitis is commonly seen across all age groups with a higher incidence in women than in men (from 3 times that of men before the age of 50 years to 1.5 times after 50-year-old). Acute cholecystitis is divided into acute calculous cholecystitis and acute noncalculous cholecystitis [5]. The onset of acute calculous cholecystitis may be attributed to bacterial infections during biliary arrest due to direct injury to the gallbladder mucosa. Acute noncalculous cholecystitis is mostly associated with severe infection or trauma, the etiology of which is still poorly understood and is mostly a local manifestation of systemic stress, i.e., severe systemic disease with severe gallbladder inflammation, mostly seen in the frail or elderly. Given the rapid onset of acute cholecystitis and its risk to *h* in severe cases, timely medical management, and hospitalization are required [6]. Currently, surgery is the mainstay of clinical treatment for acute cholecystitis to relieve the symptoms in a safe, simple, and effective manner. For elderly and frail patients, surgery should be performed with caution or elective surgery is indicated [7, 8]. Currently, laparoscopic cholecystectomy is the preferred surgical approach, in which three or four ports with a length of 0.5–1.5 cm are made in the right abdomen after the establishment of a pneumoperitoneum, followed by the opening of the triangle of Calot, severance of the cystic duct and the cystic artery, and removal of the entire gallbladder and the stones [9–11]. It is considered the gold standard for the treatment of gallstones, with significant advantages such as small trauma and rapid recovery [12]. Nevertheless, if the patient is ineligible for direct cholecystectomy, cholecystostomy or percutaneous transhepatic gallbladder drainage (PTGBD) can be performed to remove purulent bile and reduce gallbladder pressure, followed by selective cholecystectomy after stabilization of the disease. PTGBD allows rapid emptying of infected bile, reduces gallbladder tension, avoids bile duct wall rupture, decreases toxin absorption, relieves gallbladder obstruction, and controls disease progression [13]. It was found that PTGBD requires prudent use for patients with moderate acute cholecystitis due to the risk of organ damage, severe local inflammation, and the difficulty of surgical operation. In the present study, an attempt was made to assess the clinical effectiveness of laparoscopic cholecystectomy after percutaneous transhepatic gallbladder drainage (PTGBD) for acute cholecystitis so as to provide a reference for clinical treatment.

The article "Analysis of the Effect of Laparoscopic Cholecystectomy for Acute Cholecystitis after Percutaneous Transhepatic Gallbladder Puncture and Drainage" was retracted in 2023. Reasons: signs of a paper mill; compromised peer review; unreliable results or conclusions.

## 2. Materials and Methods

### 2.1. Participants

Seventy patients (32 males and 38 females, aged 25–85 years) with acute cholecystitis treated in our hospital from April 2020 to November 2021 were recruited and randomly divided into two groups of 35 patients each in order of admission (with January 2021 as the cut-off time point) to receive conventional treatment (conventional group) or PTGBD plus laparoscopic cholecystectomy (experimental group). All patients and their families gave informed and signed consent, and the study was approved by our ethics committee (Approval No.20201520).

### 2.2. Inclusion and Exclusion Criteria

#### 2.2.1. Inclusion Criteria

1. Patients who meet the clinical diagnostic criteria associated with acute cholecystitis [6].
2. Patients who are conscious and not mentally impaired.
3. Patients with an onset of more than 1 week.
4. Patients with imaging showing local adhesions, including adhesions of the gallbladder to the colon or obscure triangles of the duodenum and Calot.

#### 2.2.2. Exclusion Criteria

1. Patients with contraindications to surgery or related treatment.
2. Patients with coagulation disorders or haematological disorders.
3. Patients with a perforated gallbladder, common bile duct stones, or atrophic cholecystitis.
4. Patients with a history of upper abdominal surgery.

### 2.3. Treatment Methods

Patients in the conventional group received conventional treatment, including anti-infection, antispasmodic, analgesic, and comorbidity management, followed by laparoscopic cholecystectomy [14, 15]. After routine disinfection and draping, the patients received endotracheal intubation and general anesthesia. A CO2 pneumoperitoneum was then established with a pressure of 10–14 mm Hg. Using the conventional three or four-port laparoscopic method, laparoscopic instruments were placed through the trocars for gallbladder traction to separate the adhesions around the gallbladder and lift the hepatopancreatic ampulla. The triangle of Calot was cut open to identify the gallbladder access, common hepatic duct, and common bile duct, followed by the retrograde, antegrade, or combined dissection of the gallbladder. The gallbladder duct and gallbladder artery were severed after fixation using hemostatic clips, followed by hemostasis of the gallbladder using electrocautery, and removal of the resected gallbladder. A subhepatic drainage tube was placed for abdominal drainage and was removed 2–4 d postoperatively. In the event of serious injury to the surrounding organs that results in an unsuitable condition of the Calot's triangle for laparoscopic surgery, the patient was promptly converted to open surgery [16]. The patients received antibiotic treatment within 3–5 days after surgery.

The article "Analysis of the Effect of Laparoscopic Cholecystectomy for Acute Cholecystitis after Percutaneous Transhepatic Gallbladder Puncture and Drainage" was retracted in 2023. Reasons: signs of a paper mill; compromised peer review; unreliable results or conclusions.

Patients in the experimental group received PTGBD plus laparoscopic cholecystectomy. PTGBD was performed 40 days prior to laparoscopic cholecystectomy. After local disinfection and draping, the patient received local infiltration anesthesia with 2% lidocaine in the supine position. The condition of the gallbladder and its relationship with the surrounding organs were determined by a LOGIQE9 color Doppler ultrasound diagnostic instrument (GE, USA) using a C5-1 curved convex array probe with a probe frequency of 1–5 MHz to clarify the site of the gallbladder puncture. Cutaneous puncture was performed at the 8th or 9th intercostal space in the right axillary midline, and the puncture needle was passed through the liver tissue at the base and middle part (1/3) of the gallbladder to penetrate the gallbladder. After hollowing the needle, the purulent bile was aspirated, and the needle was then withdrawn. Along the guidewire, 4–6 cm of the deep venous catheter in the gallbladder was discarded, the guidewire was pulled out, and the catheter was attached to the skin with a sterile bag for continued voiding. In the event of poor bile flow in the catheter, the inner wall of the catheter was rinsed with 5–10 ml of saline to clear the catheter. Holistic treatment was administered during surgery, including broad-spectrum antibiotics administration, correction of water-electrolyte and acid-base imbalance, and rehydration. Postoperatively, patients received anti-infection treatment, and laparoscopic cholecystectomy was performed after 40 days, which was similar to that of the conventional group.

The serum indicator used the reagents and instruments provided by the hospital.

### 2.4. Outcome Measures

1. *Surgical Indices*. The operation time, intraoperative hemorrhage volume, time-lapse before passing gas, and hospital stay of the two groups were recorded and compared.
2. *Clinical Efficacy* [17]. The incidence of conversion to open surgery and postoperative drainage of the two groups were calculated and compared.
3. *Postoperative Recovery* [18]. The body temperature recovery time, leukocyte recovery time, and postoperative leukocyte level of the two groups were recorded and compared.
4. *Postoperative Complications* [19]. The occurrence of postoperative complications, including biliary leakage, pneumothorax, intestinal bleeding, incisional infection, respiratory failure, and liver damage, were recorded and compared between the two groups.

The article "Analysis of the Effect of Laparoscopic Cholecystectomy for Acute Cholecystitis after Percutaneous Transhepatic Gallbladder Puncture and Drainage" was retracted in 2023. Reasons: signs of a paper mill; compromised peer review; unreliable results or conclusions.

### 2.5. Statistical Analysis

The data obtained in this study were analyzed using the SPSS22.0 software. The measurement data are expressed as (mean ± standard deviation) and analyzed using the independent sample *t*-test. The count data are expressed as the number of cases (%) and tested with the chi-square test. The significance was considered statistically significant at a *P*value <less than 0.05.

## 3. Results

### 3.1. Baseline Patient Characteristics

There were 17 males and 18 females in the experimental group, aged 25–85 years, with a mean age of 60.08 ± 8.83 years, a BMI of 25.17 ± 3.63 kg/m^2^, 11 cases of diabetes mellitus, and 18 cases of hypertension. There were 15 males and 20 females in the experimental group, aged 25–85 years, with a mean age of 60.13 ± 8.21 years, a BMI of 25.37 ± 3.31 kg/m^2^, 9 cases of diabetes mellitus, and 21 cases of hypertension. The baseline patient characteristics of the two groups were comparable (*P* > 0.05) (Table 1).

### 3.2. Surgical Indices

Patients in the experimental group were associated with significantly less intraoperative hemorrhage volume and shorter operative time, time-lapse before passing gas, and hospital stay (83.15 ± 31.17, 32.54 ± 12.61, 23.02 ± 4.61, 7.98 ± 3.24) versus those in the conventional group (120.56 ± 30.55, 61.01 ± 15.54, 28.15 ± 5.91, 11.95 ± 4.15) (*P* < 0.05) (Table 2).

### 3.3. Clinical Efficacy

The incidence of conversion to open surgery and postoperative drainage in the experimental group was significantly lower (2.86%, 5.71%) than that of the conventional group (25.71%, 45.71%) (*P* < 0.05) (Table 3).

### 3.4. Postoperative Recovery

The differences in the postoperative body temperature of the two groups did not come up to the statistical standard (*P* > 0.05). The experimental group had faster body temperature recovery and leukocyte recovery and better leukocyte levels (1.25 ± 0.56, 2.36 ± 0.48, 7.92 ± 1.36) than the conventional group (3.11 ± 1.05, 5.41 ± 0.63, 10.52 ± 2.78) (*P* < 0.05) (Table 4).

The article "Analysis of the Effect of Laparoscopic Cholecystectomy for Acute Cholecystitis after Percutaneous Transhepatic Gallbladder Puncture and Drainage" was retracted in 2023. Reasons: signs of a paper mill; compromised peer review; unreliable results or conclusions.

### 3.5. Complications

In the experimental group, there was 1 (2.86%) case of pneumothorax and 1 (2.86%) case of intestinal bleeding. In the conventional group, there were 2 (5.71%) cases of biliary leakage, 3 (8.57%) cases of pneumothorax, 4 (11.43%) cases of intestinal bleeding, 5.71% cases of incisional infection, 1 (2.86%) case of respiratory failure, and 1 (2.86%) case of liver damage. The experimental group showed a significantly lower incidence of complications (5.71%) versus the conventional group (37.14%) (*P* < 0.05) (Table 5).

## 4. Discussion

Cholecystitis is the collective term for acute cholecystitis and chronic cholecystitis and refers to a process of acute or chronic inflammatory reaction in the gallbladder caused by gallbladder stones [20]. Cholecystitis is a common surgical disease with high prevalence and is divided into acute and chronic types according to its clinical manifestations. In the acute phase of cholecystitis, the symptoms of epigastric pain can be severe and the disease progresses rapidly, which requires urgent medical attention. Chronic cholecystitis often coexists with gallbladder stones and compromises the quality of life of patients despite mild symptoms [9]. Routine treatment of cholecystitis primarily focuses on aggressive prevention and treatment of bacterial infections and complications. In chronic cholecystitis, symptomatic antispasmodic, analgesic, and anti-inflammatory treatment, together with daily dietary care, deserve great attention [21]. In the case of acute cholecystitis, laparoscopic cholecystectomy is the main treatment for cholecystitis. However, the unclear anatomical plane of Calot's triangle in acute cholecystitis leads to difficulties in gallbladder separation, which prevents the direct implementation of laparoscopic cholecystectomy. Moreover, cholecystitis develops rapidly with severe complications, heavily compromising the health and safety of patients. Clinical treatment of acute cholecystitis targets symptom relief, elimination of infection, and drainage of stagnant bile, for which conservative therapy is mostly adopted to stabilize patient condition prior to surgical interventions. However, as summarized by years of clinical practice, conservative therapy is considered unsatisfactory [22, 23]. PTGBD, as an alternative to cholecystostomy, facilitates decompression of the patient's gallbladder to achieve adequate drainage, relieve obstruction, and alleviate clinical symptoms [24]. It features multiple merits, such as simple operation, low price, high safety, and reliability, and it minimizes the trauma to the gallbladder wall with little impact on the patient's systemic condition.

The article "Analysis of the Effect of Laparoscopic Cholecystectomy for Acute Cholecystitis after Percutaneous Transhepatic Gallbladder Puncture and Drainage" was retracted in 2023. Reasons: signs of a paper mill; compromised peer review; unreliable results or conclusions.

The results of the present study showed that patients in the experimental group showed significantly less intraoperative hemorrhage volume and shorter operative time, time-lapse before passing gas, and hospital stay versus those in the conventional group, and the incidence of conversion to open surgery and postoperative drainage of the experimental group was significantly lower than that of the conventional group (*P* < 0.05), suggesting significant benefits of PTGBD following laparoscopic cholecystectomy for patients with acute cholecystitis. The reason may be that compared with direct surgery after conventional therapeutic intervention, PTGBD allows for a better surgical condition and reduces the operation time and intraoperative bleeding. Prior studies revealed that most patients had missed the optimal 72-hour surgery window by the time of admission, and intraoperative adhesions around the gallbladder and the Calot's triangle were observed, resulting in difficulty in dissection and separation under laparoscopy and a higher incidence of intraoperative conversion to open surgery. In the present study, PTGBD treatment significantly reduces bile duct pressure and gallbladder edema, improves surgical outcomes, and reduces surgical risk. The results were in accordance with the previous research results. Moreover, the differences in the postoperative body temperature of the two groups did not come up to the statistical standard (*P* > 0.05), and the experimental group had faster body temperature recovery, leukocyte recovery, and better leukocyte levels than the conventional group (*P* < 0.05), which may be attributable to the fact that PTGBD promptly relieves biliary pressure in patients and significantly mitigates their clinical symptoms, and local anesthesia has little effect on the recovery of the patient [25]. Furthermore, the experimental group showed a significantly lower incidence of complications (5.71%) versus the conventional group (37.14%) (*P* < 0.05), indicating that PTGBD prior to laparoscopic cholecystectomy constitutes a viable alternative for the treatment of acute cholecystitis, which is attributable to the increased patient tolerance to surgery after the amelioration of patient conditions by performing PTGBD [13]. The results are in line with the findings of Tan et al. (2018), whose study demonstrated that PTGBD could lower the risk of postoperative complications in acute cholecystitis in the elderly, effectively shorten the operative time and postoperative hospital stay, and reduce intraoperative bleeding [26].

Chronic cholecystitis requires symptomatic antispasmodic, analgesic, and anti-inflammatory treatments, as well as attention to daily diet [27]. Antispasmodic and analgesic drugs, such as atropine or demerol, are available for severe upper abdominal pain in the acute phase [28]. Furthermore, timely antibacterial treatment, such as ampicillin, clindamycin, and aminoglycosides, is also required [29]. In addition, choleretic drugs, such as magnesium sulfate, are also encouraged to potentiate the treatment efficiency [30]. For patients with cholecystitis, anti-inflammatory and choleretic Chinese patent medicines, such as Jindan Tablets or Qinggan Lidan Oral Liquid can also be used daily to promote the discharge of bile and reduce the inflammation of the gallbladder [31]. In Chinese medicine, moxibustion and acupuncture are considered effective adjunctive treatments to invigorate the blood and alleviate the clinical symptoms of patients [32]. External drug treatment also contributes to the mitigation of the inflammation of the gallbladder to mitigate the symptoms [33].

The article "Analysis of the Effect of Laparoscopic Cholecystectomy for Acute Cholecystitis after Percutaneous Transhepatic Gallbladder Puncture and Drainage" was retracted in 2023. Reasons: signs of a paper mill; compromised peer review; unreliable results or conclusions.

However, there are several limitations to this study. Firstly, this study was conducted on a small group of patients from our hospital and might result in bias. Secondly, a follow-up trial was absent to determine prognosis and long-term effects. Future studies with a long-term follow-up and analysis of the molecular mechanisms will be conducted to provide more reliable data.

## 5. Conclusion

PTGBD plus laparoscopic cholecystectomy for acute cholecystitis effectively improves surgical safety, promotes patients' postoperative recovery, and reduces the incidence of conversion to open surgery and postoperative complications with a high safety profile. Further trials are, however, required prior to clinical promotion.

## Figures and Tables

**Table 1:** Baseline patient characteristics ($\bar{x}\pm s$).

Group	*n*	Gender		Age (year)		BMI (kg/m^2^)	Underlying disease	
		Male	Female	Range	Mean		Diabetes mellitus	Hypertension
Experimental	35	17	18	25–85	60.08 ± 8.83	25.17 ± 3.63	11	18
Conventional	35	15	20	25–85	60.13 ± 8.21	25.37 ± 3.31	9	21
*t*	—	—	—	—	0.025	0.241	—	—
*P value*	—	—	—	—	0.980	0.810	—	—

**Table 2:** Surgical indices ($\bar{x}\pm s$).

Group	*n*	Operative time (min)	Intraoperative hemorrhage volume (ml)	Time-lapse before passing gas (h)	Hospital stay (d)
Experimental	35	83.15 ± 31.17	32.54 ± 12.61	23.02 ± 4.61	7.98 ± 3.24
Conventional	35	120.56 ± 30.55	61.01 ± 15.54	28.15 ± 5.91	11.95 ± 4.15
*t*	—	5.071	8.416	4.049	4.461
*P value*	—	<0.001	<0.001	<0.001	<0.001

**Table 3:** Conversion to open surgery and postoperative drainage (%).

Group	*N*	Conversion to open surgery		Postoperative drainage	
		*n*	Rate	*n*	Rate
Experimental	35	1	2.86	2	5.71
Conventional	35	9	25.71	16	45.71
*x* ^*2*^	—	7.467		14.658	
*P value*	—	0.006		<0.001	

The article "Analysis of the Effect of Laparoscopic Cholecystectomy for Acute Cholecystitis after Percutaneous Transhepatic Gallbladder Puncture and Drainage" was retracted in 2023. Reasons: signs of a paper mill; compromised peer review; unreliable results or conclusions.

**Table 4:** Postoperative recovery ($\bar{x}\pm s$).

Group	*N*	Recovery time		Postoperative level	
		Body temperature (d)	Leukocyte (d)	Body temperature (°)	Leukocyte (×10^9^/L)
Experimental	35	1.25 ± 0.56	2.36 ± 0.48	37.88 ± 0.62	7.92 ± 1.36
Conventional	35	3.11 ± 1.05	5.41 ± 0.63	38.01 ± 0.74	10.52 ± 2.78
*T*	—	9.247	22.782	0.797	4.97
*P value*	—	<0.001	<0.001	0.428	<0.001

**Table 5:** Postoperative complications (%).

Group	*N*	Biliary leakage	Pneumothorax	Intestinal bleeding	Incisional infection	Respiratory failure	Liver damage	Total incidence
Experimental	35	0 (0.00)	1 (2.86)	1 (2.86)	0 (0.00)	0 (0.00)	0 (0.00)	2 (5.71)
Conventional	35	2 (5.71)	3 (8.57)	4 (11.43)	2 (5.71)	1 (2.86)	1 (2.86)	13 (37.14)
*x* ^*2*^	—	10.267						
*P value*	—	0.001						

## Data Availability

All the data used in this study are shown in figures and tables.
